# Design of IoT Gateway for Crop Growth Environmental Monitoring Based on Edge-Computing Technology

**DOI:** 10.1155/2022/8327006

**Published:** 2022-07-14

**Authors:** Mo Dong, Haiye Yu, Zhipeng Sun, Mingzhi Wu, Lei Zhang, Yuanyuan Sui, Guanghao Yu, Ting Han, Ruohan Zhao

**Affiliations:** ^1^College of Biological and Agricultural Engineering, Jilin University, Changchun 130022, Jilin, China; ^2^Mudanjiang Medical University, Mudanjiang 157000, Heilongjiang, China; ^3^Nanchang Automotive Institution of Intelligence & New Energy, Nanchang 330052, Jiangxi, China

## Abstract

With the extensive use of the Internet of Things (IoT) in agriculture, the number of terminals are also grow rapidly. This will increase the network traffic and computing pressure of the centralized server. The centralized data processing mode used in traditional agriculture cannot meet the needs of the Internet of everything era. This paper designs a gateway based on edge-computing technology for monitoring crop growth environment. It uses virtualized container technology to package long-range wide-area network (LoRaWAN) server, pest identification, and environmental information data fusion functions into images. It forms integrated operation mode of multiple function in agriculture. The gateway applies message-oriented middleware to standardize and customize the data transmission among functional modules, clouds, and edges. Through simulation and field test, the designed gateway can achieve the functions of each module at the same time, the resource utilization, and the transmission quality are stable. The edge-computing gateway has the advantages of low cost, low latency, and low power consumption which has practical significance.

## 1. Introduction

With the rapid development of Internet of Things (IoT) technology in agriculture, the monitoring of the growth environment of crops can obtain real-time information such as water and fertilizer using, diseases, and pests. These data can be fed back and analyzed by expert to guide production. However, due to the extensive use of the IoT in agriculture, the number of terminals are also grow rapidly which will increase the network traffic and computing pressure of the centralized server. The centralized data processing mode used in traditional agriculture cannot meet the needs of the Internet of everything era. The emergence of edge computing means that many tasks such as identification of pests and analysis of a large amount of agricultural field data that used to require cloud processing can be implemented locally. Edge-computing technology can greatly increase the response speed of agricultural information, improve the monitoring accuracy, and formulate production strategies for monitoring areas more effectively.

In edge-computing technology, downstream data represents cloud center, upstream data represents interconnected services, and the edge refers to computing and network resources from the data source to the cloud center [1]. Edge computing can calculate, store, and apply the data uploaded by nodes near the source and provide real-time processing services. It can meet the requirements of online real-time data processing, safe transmission, and decision-making in intelligent agriculture [2, 3].

Although the edge-computing technology has made great progress in the application of IoT, still this opens up research questions:(1). Edge-computing technology is rarely used in the agricultural IoT, especially when the gateway accesses different types of agricultural data at the same time. (2) Edge-computing technology combined with container technology in the field of agricultural IoT is also basically in the initial stage. (3) The research on cloud-edge architecture and online algorithm of IoT applied to crop growth environmental monitoring is still in the blank stage.

To underpin the relevance of the research questions, the following are the contributions of this paper:

- We design an IoT gateway for crop growth environmental monitoring based on edge-computing technology which includes both function and communication architecture.
- We use virtualized container technology to package LoRaWAN server, pest identification, and environmental information data fusion functions into images which form integrated operation mode in agriculture.
- We apply message-oriented middleware to standardize and customize the data transmission among functional modules, clouds, and edges in the gateway which reduces the pressure of cloud computing, lowers the transmission delay between cloud and edge.

This paper is outlined as follows.  Section 2 gives related work of applications of edge-computing and docker technology.  Section 3 describes the design of edge-computing gateway framework.  Section 4 provides the experimental results and performance evaluation include transmission stability of LoRaWAN server, stress testing of Message Queuing Telemetry Transport (MQTT) message-oriented middleware, stability test of edge-computing architecture, and field test.  Section 5 summarizes our contributions and prospects, concludes this article.

## 2. Related Works

The research on edge computing began in 1998, Akamai Company designed a content delivery network (CDN) system based on distributed cache server. The system accomplished load balancing, computing scheduling, and data forwarding operations for each distributed cache server through the master server. This improved the response speed and connection success rate of user accessing to the server [4]. In 2009, Satyanarayanan et al. introduced the concept of Cloudlet. It used fixed computing resources closer to clients to increase computing power of traditional cloud servers. The scheme focused on the downlink capability of edge computing, moved some cloud server functions to the edge and further reduced bandwidth consumption and latency. Since then, with the development of the IoT and mobile communication technology, more attention has been paid to the data processing, transmission, and storage of edge computing. This paper summarizes applications of the edge-computing technology in recent years and analyzes their advantages as shown in Table 1.

How to dynamically match computing resources in heterogeneous computing environment to optimize system performance is a challenge for edge-computing field.

In the case of applying edge-computing technology in IoT, application of small board equipment with low cost and limited resources are becoming more and more popular. The virtualization technology applied to small board devices can ensure the implementation of some cloud computing tasks on devices of edge computing, and it has good flexibility and scalability [13–16]. Virtualization technology enables users to make full use of resources by transforming physical resources such as networks, computing, storage so that services are no longer limited by hardware [17]. As a virtualization technology, container has been widely used in resource management, system maintenance, and software deployment of cloud computing platforms in recent years. It is also gradually applied to edge computing. Docker is a container engine based on Linux kernel virtualization technology. It was developed using GO language and apache2.0 protocol and was released on GitHub in 2013. Docker uses Cgroups technology to manage process resources and uses namespace to isolate system resources. While providing isolation, the container can also achieve resource sharing [18]. Compared with traditional virtual machines, Docker starts quickly, deploys easily, and uses less resources [19]. However, the application of real-time container technology is often not considered in edge computing at this stage.

## 3. Proposed Edge-Computing Gateway Framework

### 3.1. Design of Edge-Computing Gateway

Gateway is a computer system or device that converts between networks with different communication protocols and data structures. IoT gateway is the core component, and it is the bridge between the terminal nodes and the cloud. This paper designs an edge-computing gateway, and it is the regional network information center of crop growth environmental monitoring IoT. The edge-computing gateway provides a layer with communication and data processing capabilities between the terminal devices and the cloud server. This structure has good performance in transmission delay and stability, as shown in Figure 1.

In this paper, we combine the situation of environmental monitoring with the functional view of edge computing and design the architecture of edge-computing gateway. The architecture is divided into data access layer, virtualization layer, and function layer. This architecture enables all kinds of situations in agricultural applications to be analyzed and processed quickly. The architecture is shown in Figure 2.

#### 3.1.1. Data Access Layer

The data access layer of the edge-computing gateway supports a variety of hardware interfaces and bus protocols. We customize LoRaWAN and Wi-Fi protocols and equip with communication module. Through the multithreading technology of Linux system, the drivers can be called concurrently. This ensures the real-time data transmission and provides data support for edge computing.

#### 3.1.2. Virtualization Layer

We use Docker as the virtualization platform. The containerized architecture can split the original services that need to be performed on cloud servers. It also provides a clear boundary between different services through isolation technology. This can make better use of the hardware computing resources. Base on Docker virtualization technology, services that need to run independently are packaged into images. In this way, each service is isolated from each other. The virtual network provides data access services for the container, and it improves the resource utilization efficiency and compatibility of the edge-computing gateway.

#### 3.1.3. Functional Layer

The function layer defines the input and output of each function container by managing the images. This layer processes data uploaded by terminal nodes and achieves cloud functions at the edge. The main functions of our design include pest identification, crop growth environmental information monitoring and processing, and integration of LoRaWAN server. In addition, we also retain the functional interfaces, and this will provide resources for the customized services according to the requirements of the agricultural IoT.

### 3.2. Main Functional Modules of Edge-Computing Gateway

#### 3.2.1. MQTT Service Module

Docker container completes data transmission through virtual network interface. The virtual network communication between containers uses the data exchange method of Linux kernel. Virtual network interface reduces the time loss caused by the transmission of physical network devices. Data packets are directly transmitted and exchanged within the processor. Although the containers can be accessed through Docker bridge, the traditional interaction mode between containers is generally using IP address, which has the problems of complex interaction and poor expansibility.

In this paper, we use the MQTT message-oriented middleware and apply the publish/subscribe mode to complete message transmission. The principle is shown in Figure 3. In this design, message-oriented middleware is also applied to data interaction between edge-computing gateway and cloud. At present, most of Internet architectures support MQTT protocol. The MQTT Broker has become a bridge for information exchange in the cloud-edge architecture.

In this design, RabbitMQ developed by Rabbit Technology Co., Ltd. is used as the software carrier of MQTT message-oriented middleware. RabbitMQ is written in Erlang language. It completes asynchronous message processing through advanced message queuing protocol. RabbitMQ supports cluster operation and has good flexibility and scalability. The RabbitMQ structure is shown in Figure 4.

#### 3.2.2. LoRaWAN Server Module

Under the traditional LoRaWAN architecture, LoRaWAN server is generally installed in the cloud. The cloud communicates with the field gateway through the wireless Internet, and it is greatly affected by the quality of the field network. Once the gateway loses the Internet, the entire IoT system will not work. Moreover, the frequent communication between the gateway and the cloud will also lead to excessive consumption of bandwidth resources and transmission delay. In this design, LoRaWAN server is installed in the edge-computing gateway. However, if the LoRaWAN server is directly installed in the Linux system, due to the complex structure, it will occupy more memory, processes, and interfaces. This will reduce the data processing capacity of the entire edge-computing gateway. Through container technology, we isolate the LoRaWAN server into a separate container. Based on Docker's excellent isolation technology, it can achieve complete LoRaWAN service support at the gateway.

#### 3.2.3. Pest Identification Module

With the increase of high-quality images transmission on the Internet, the delay of cloud computing is significantly higher than that of edge computing. The main function of this module is to monitor, collect, transmit, and process the pests image in farmland. The module uses Python language to write pest identification and counting algorithm based on deep learning, achieves the identification, counting, and other processing of the pest images collected by the monitoring nodes.

#### 3.2.4. Crop Growth Environmental Information Monitoring Module

The main function of this module is to monitor, collect, transmit and process the environmental information of farmland. The information includes seven different environmental factors: light intensity, air temperature, air humidity, soil humidity, soil temperature, CO_2_ concentration, and soil conductivity. This module collects and transmits the information of various sensors arranged in the farmland to the gateway. Data processing and fusion algorithms are designed and used at the edge to improve the measurement accuracy. The module is written in Python language, using Python scientific computing library Numpy, and data analysis package Pandas. The data fusion algorithm of this module is as follows:

In the process of sensors acquiring data, the measured value *X*_*i*_, the true value *Z*_*i*_ and the noise value *Y*_*i*_ of the sensor have the relationship of equation:

(1) $$\begin{array}{c} X_{i}=Z_{i}+Y_{i}\left(i=1,2,\ldots ,n\right). \end{array}$$

The following steps are taken to reduce noise error:

(1) Sort the data collected by all sensors and select the maximum value *X*_max_ and the minimum value *X*_min._
(2) Take the average *A*_0_ of the maximum and minimum values obtained.
  (2) $$\begin{array}{c} A_{0}=\frac{X_{\max}+X_{\min}}{2}. \end{array}$$
(3) Add the obtained average *A*_0_ to the original data and rearrange them. At this time, the part greater than or equal to *A*_0_ is classified as *P*_1_, and the part less than *A*_0_ is classified as *P*_2._
  (3) $$\begin{array}{c} \left\{\begin{array}{c} P_{1}=\left[X\left(n\right)|X\left(n\right)\geq A_{0}\right]\\ P_{2}=\left[X\left(n\right)|X\left(n\right)\geq A_{0}\right] \end{array}\right\}. \end{array}$$
(4) Continue to calculate the average value of *P*_1_ and *P*_2_. After obtaining *P*_1*a*_ and *P*_2*a*_, average them again
  (4) $$\begin{array}{c} A_{1}=\frac{P_{1a}+P_{2a}}{2}. \end{array}$$
(5) Add the obtained average value *A*_*1*_ to the original data again, repeat the above steps until equation (5) is satisfied, and stop the iteration:
  (5) $$\begin{array}{c} A_{k}=A_{k-1}. \end{array}$$

At this time, the average value obtained is no longer changed, and it is considered that the value is infinitely close to the real data.

### 3.3. Workflow of Edge-Computing Gateway

#### 3.3.1. Data Access of Terminal Nodes

*(1) Data Access of Environmental Monitoring Nodes*.

The environmental information monitoring data from the terminal sensor communicates with the LoRaWAN server in the following ways: Packet Forwarder (PF) is a program running on the host of LoRa gateway, which is mainly responsible for data message forwarding between the terminal and LoRaWAN server. PF forwards the data packets uploaded by the environmental monitoring nodes to the LoRaWAN server module in the form of UDP packets. LoRaWAN server performs packets decryption, forwarding, and other operations. Similarly, PF converts the downlink medium access control (MAC) commands and other data of LoRaWAN server into Radio Frequency (RF) packets and sends them to the environmental monitoring nodes, as shown in Figure 5.

*(2) Data Access of Pest Identification Nodes*.

The edge-computing gateway uses Wi-Fi to communicate with the pest monitoring nodes and obtains the images by establishing a socket connection. The images uploaded through Wi-Fi are converted into image coding by OpenCV and temporarily stored in the specific path of the module. We use the script to regularly check whether there are updates under the path. If there is a new image, the pest recognition processing will be performed. After image preprocessing and identification, the current number and species of pests will be transmitted to cloud through MQTT protocol. The data access of pest identification nodes is shown in Figure 6.

#### 3.3.2. Message-Oriented Middleware Service

In this design, we build message-oriented middleware transmission architecture with MQTT Broker as the hub. The communication between each module uses the push mode with unique “topic” subscription. The topics used in this design are shown in Table 2. The transmission architecture is shown in Figure 7.

The interface of RabbitMQ is shown in Figure 8. After building an image through Docker, we can view the user's status on the page after the device is connected. RabbitMQ as an MQTT server is responsible for message forwarding through topics and saving logs.

#### 3.3.3. Management of Docker

In this design, Docker container is used to isolate the functional modules of edge-computing gateway. The internal communications between containers are carried out in the form of independent services, and each container provides necessary interfaces. The LoRaWAN server, environmental monitoring, pest identification, and other functional modules in the edge-computing gateway are all running in the mode of virtual container. From the perspective of hardware resources, each virtualization service container allocates resources through Docker. This enables more rational use of CPU computing power, data storage, and other resources. Docker is convenient for function splitting and reorganization, and we can manage a container by using commands alone, or use Docker compose (a tool for batch container management) for batch processing. The process is shown in Figure 9.

### 3.4. Hardware of Edge-Computing Gateway

We choose Raspberry Pi 4b as the hardware of the edge-computing gateway. Raspberry Pi is a single-board microcomputer with ARM processor architecture, low-power consumption, and high performance. Its CPU uses ARM Cortex-A72 1.5 GHz (quad core) processor and supports 64-bit operation. Raspberry Pi has 8 GB of running memory and Wi-Fi module, supports 5 GHz and 2.4 GHz under 802.11 g. It also supports microSD card, serial port, and GPIO communication. Raspberry Pi carries 4G transmission module through USB interface to exchange data with cloud. Although the size is similar to a hand, it can complete most of the processing task of a computer. With the support of hardware interface and external network module, it has the ability to achieve edge-computing tasks. Photo of edge-computing gateway based on Raspberry Pi is shown in Figure 10.

## 4. Experimental Results and Analysis

### 4.1. Transmission Stability of LoRaWAN Server

In order to better verify the data transmission stability of LoRaWAN server in an edge-computing gateway, this paper builds a simulation system of LoRaWAN transmission quality based on ns-3 software using Ubuntu 16.04 OS. ns-3 simulation software, developed in 2006, it is an open-source network simulation software driven by discrete events. ns-3 is mainly used to simulate wireless transmission networks. In this simulation, we choose eight common data transmission intervals of agricultural IoT. In addition, in order to test the stability of concurrent data transmission of multiple monitoring nodes and gateways, we set the number of environmental monitoring nodes to 0–1000 and the number of edge-computing gateways to 1, 2, and 4. We divide the sending data into two types: with acknowledgment (ACK) and without ACK. For the transmission stability between the crop growth environmental monitoring nodes and LoRaWAN server, we conduct the following tests.

#### 4.1.1. Single Gateway

*(1) Relationship between Transmission Interval and Packet Loss Rate*.

In this simulation, we choose a single edge-computing gateway, set the transmission interval as 60, 120, 200, 400, 600, 800, 1000, and 1200 s, and fix the number of environmental monitoring nodes at 200. We divide the sending data into two types: with ACK and without ACK. The relationship between packet loss rate and transmission interval is shown in Figure 11.

*(2) Relationship between the Number of Nodes and Packet Loss Rate*.

In this simulation, we choose a single edge-computing gateway, and transmission interval is fixed at 600 s. The relationship between the number of environmental monitoring nodes (0–1000) and the packet loss rate is shown in Figure 12.

#### 4.1.2. Multi Gateway

*(1) Relationship between the Number of Nodes and Packet Loss Rate*.

In this simulation, we choose 1, 2, and 4 gateways separately, and the transmission interval is fixed at 600 s. We also divide the sending data into two types: with ACK and without ACK. Figures 13 and 14 show the relationship between the number of environmental monitoring nodes (0–1000) and the packet loss rate.

#### 4.1.3. Result Analysis

1. It can be seen from Figure 11 that with the gradual increase of transmission interval, whether the transmission has ACK or not, the packet loss rate will gradually decrease. When the data transmission interval is once a minute, the packet loss rate still be controlled less than 5%. In the field of communication, it is generally believed that when the packet loss rate is less than 5%, the communication quality is good. Therefore, it meets the requirements of transmission quality.
2. From Figure 12, we can see that with the increase of the number of monitoring nodes, the packet loss rate of both transmission modes increase, and it is the same as expected. However, even when the number of monitoring nodes reaches 1000, the packet loss rate remains at a low level (less than 5%). Therefore, it also meets the requirements of transmission quality.
3. From Figures 13 and 14, we can see that using multigateways at the same time will not affect the quality of transmission. This further shows that using multiple gateways with LoRaWAN server can expand the monitoring area of farmland without reducing the transmission quality.
4. By analyzing Figures 11–14, we can know that whether the transmission with ACK is used or not, the packet loss rate is less than 5%. There is little difference between the two transmission modes. The specific advantages of the two transmission modes need further simulation analysis, which will not be discussed in this paper.

Through the above analysis, we can conclude that installing LoRaWAN server on the edge-computing device can effectively increase the transmission distance and the monitoring range of farmland. At the same time, the data transmission is stable and meets the transmission quality requirements. This provides an effective method for future research on long-distance transmission and larger area of farmland environmental monitoring.

### 4.2. Stress Testing of MQTT Message Oriented Middleware

#### 4.2.1. Research Methods

Information forwarding capability is an important performance of edge-computing gateway. Information forwarding capabilities are mainly reflected in the success rate of sending messages, delaying situation, and other information forwarding statistics. We use a concurrent stress testing that sends 1–1000 data per second to test the success rate and delaying situation of message-oriented middleware when processing data.  Figure 15 shows the packet loss rate of message forwarding at the frequency of 1–1000 messages per second.

#### 4.2.2. Result Analysis

The test results show that the gateway's information forwarding capability is stable. Under the stress testing of 1000 concurrent messages, the packet loss rate is about 2%. It meets the requirements of transmission quality.

In farmland environmental monitoring, the frequency of data transmission usually does not reach the state of stress testing. This shows the transmission mechanism based on MQTT message-oriented middleware can be well applied to the edge-computing gateway.

### 4.3. Stability Test of Edge-Computing Architecture

#### 4.3.1. Research Methods

In operation and maintenance, we often use the average load to represent the average number of processes in the running state and noninterruptible state of the system. This is also a measurement parameter to characterize the overall operation state of the system. Average load is closely related to the number of CPU cores in the hardware. If the average load is more than the number of CPU cores, the system is considered to be in an overloaded state, which will affect all processes of the system, causing the system to run slowly or even crash.

In this design, the Raspberry Pi adopts a quad core processor that supports 64-bit operation. By monitoring the average gateway load during the stress testing, we can see the gateway's average load and memory usage under 500/1000 concurrent messages per second as shown in Figures 16 and 17.

#### 4.3.2. Result Analysis

Under the stress testing of 500 concurrent messages per second, the average load of the gateway is 0.22, while with 1000 concurrent messages per second, the average load of the gateway is 2.99, which are both less than the number of CPU cores. The above experiments show that the gateway works stably and reliably in stress testing.

Through the test, we can see that the edge-computing gateway architecture based on Raspberry Pi fully meets the complex state requirements of high-speed data transmission, which provides a new method for the application of mobile edge-computing technology.

### 4.4. Field Test of Edge-Computing Gateway

We also carried out field tests in the Siping area of Jilin Province in China. The nodes of the pest identification module and the environmental monitoring module both uploaded a set of data per minute. The results showed that all the modules are working stably. A through checking of information sent and received by the cloud network within 48 hours, the environmental monitoring nodes sent 8640 messages and the pest identification nodes sent 2880 messages. The cloud received 8572 and 2845 messages, and the success rates were 99.21% and 98.78%, respectively. The average success rate of was 99.1%, as shown in Table 3.

## 5. Conclusion and Prospects

### 5.1. Conclusion

This paper designs an IoT gateway for crop growth environmental monitoring based on edge-computing technology. According to the characteristics of online monitoring data transmission, the Gateway uses virtualized container technology to package LoRaWAN server, pest identification, and environmental information data fusion functions into images. And it forms integrated operation mode of multiple function in agricultural field. The gateway applies message-oriented middleware to standardize and customize the data transmission among function modules, clouds, and edges.

The simulation result shows that the data transmission based on LoRaWAN protocol is stable. The packet loss rate is less than 5% and meets the transmission quality requirements. The gateway can achieve the functions of each module at the same time. In the stress testing of 500/1000 concurrent data per second, the average load is 0.22/2.99, and the system resource utilization is stable. In the field test, the average success rate of data transmission is 99.1%.

In this paper, the heterogeneous integration of two transmission protocols of LoRaWAN and Wi-Fi is used in farmland environmental monitoring for the first time. From the aspect of computing power distribution, functional modules such as pest identification and data fusion are equipped at the edge which can process the information uploaded by the terminal nodes in real-time. The edge-computing gateway reduces the pressure of cloud computing, lowers the transmission delay between cloud and edge. Also, it reduces the occupation rate of network bandwidth resources and further improves the transmission efficiency. In summary, the edge-computing gateway we designed has the advantages of low cost, low latency, and low power consumption compared with similar devices which has practical significance.

### 5.2. Prospects

Although this paper has done some actual work on the establishment of gateway based on edge-computing technology and conducted tests, there are still some problems to be solved. For example, when the monitoring range of farmland is very large, Wi-Fi transmission will be limited. How to combine 5G technology will be the research object in future. In addition, there are other two research axes we wish to develop: (1) Further improve the designed edge-computing gateway and add more module functions, such as automatic control module, so as to study the automatic control system of water and fertilizer. (2) Continue to do research on agricultural IoT, we are going to apply the edge-computing gateway to the large-scale farmland environmental monitoring system and form a regional grid. At the same time, combined with the cloud platform, make it become an important part in intelligent agriculture.

## Figures and Tables

**Figure 1:** Relationship between cloud, edge-computing layer, and terminal.

**Figure 2:** Architecture of edge-computing gateway.

**Figure 3:** Diagram of message-oriented middleware.

**Figure 4:** Structure of RabbitMQ.

**Figure 5:** Data access process of environmental monitoring nodes.

**Figure 6:** Data access process of pest identification nodes.

**Figure 7:** Transmission architecture of edge-computing gateway based on MQTT.

**Figure 8:** Interface of RabbitMQ.

**Figure 9:** Management of docker container.

**Figure 10:** Photo of edge-computing gateway based on raspberry Pi.

**Figure 11:** Relationship between transmission interval and packet loss rate under single gateway.

**Figure 12:** Relationship between the number of nodes and packet loss rate under single gateway.

**Figure 13:** Relationship between the number of nodes and packet loss rate under multigateway (without ACK).

**Figure 14:** Relationship between the number of nodes and packet loss rate under multigateway (with ACK).

**Figure 15:** Packet loss rate under the condition of 1–1000 concurrent data per second.

**Figure 16:** Average load under 500 concurrent messages per second.

**Figure 17:** Average load under 1000 concurrent messages per second.

**Table 1:** Literature review of edge-computing applications.

Literature	Application scenarios	Advantage			
		Security	Low cost	Low latency	Low power consumption
[5]	Finding nodes of Internet of things				✓
[6]	Traceability of shipyard pipeline processing			✓	
[7]	Detection of industrial thermal anomaly			✓	
[8]	Manufacturing architecture of decision-making		✓	✓	
[9]	Encryption of smart grid data	✓			
[10]	Networked control of industrial robots		✓	✓	
[11]	Application of machine learning in industry	✓		✓	
[12]	A smart IoT monitoring based on UAV		✓	✓	

**Table 2:** Topic description of message-oriented middleware.

Topic name	Producer	Consumer	Description
LoRAWAN	LoRaWAN server	Data fusion processing module	Data uploaded by environmental monitoring sensors
Pest identification	Pest identification module	Cloud server	Data uploaded by pest identification module nodes
Data fusion	Data fusion processing module	Cloud server	Environmental information data processed by data fusion processing module

**Table 3:** Success rate of sending and receiving data within 48 hours.

Data source	Number of sent messages	Number of received messages	Success rate（%）
Environmental monitoring nodes	8640	8572	99.21
Pest identification nodes	2880	2845	98.78
Total data	11520	11463	99.10

## Data Availability

The data used to support the findings of this study are available from the corresponding author upon request.
